The article "The Identification and Clinical Value Evaluation of CYCS Related to Asthma through Bioinformatics Analysis and Functional Experiments" was retracted in 2023. Reasons: signs of a paper mill; compromised peer review; unreliable results or conclusions.

# The Identification and Clinical Value Evaluation of CYCS Related to Asthma through Bioinformatics Analysis and Functional Experiments

**DOI:** 10.1155/2023/5746940

**Published:** 2023-04-14

**Authors:** Yan Li, Li Li, Hua Zhao, Xiwen Gao, Shanqun Li

**Affiliations:** ^1^Department of Pulmonary Medicine, Minhang Hospital, Fudan University, 170 Xinsong Road, Shanghai, China 201199; ^2^Department of Pulmonary Medicine, Zhongshan Hospital, Fudan University, 180 Fenglin Road, Shanghai, China 200032

## Abstract

**Background:**

Asthma is one of the most common respiratory diseases and one of the largest burdens of health care resources across the world. This study is aimed at using bioinformatics methods to find effective clinical indicators for asthma and conducting experimental validation.

**Methods:**

We downloaded GSE64913 data and performed differentially expressed gene (DEG) screening. Weighted gene coexpression network analysis (WGCNA) on DEGs was applied to identify key module most associated with asthma for protein-protein interaction (PPI) analysis. According to the degree value, ten genes were obtained and subjected to expression analysis and receiver operating characteristic (ROC) analysis. Next, key genes were screened for expression analysis and immunological analysis. Finally, cell counting kit-8 (CCK-8) and qRT-PCR were also conducted to observe the influence of hub gene on cell proliferation and inflammatory cytokines.

**Results:**

From the GSE64913 dataset, 711 upregulated and 684 downregulated DEGs were found. In WGCNA, the top 10 genes in the key module were examined by expression analysis in asthma, and CYCS was determined as an asthma-related oncogene with a good predictive ability for the prognosis of asthmatic patients. CYCS is significantly associated with immune cells, such as HHLA2, IDO1, TGFBR1, and CCL18 and promoted the proliferation of asthmatic cells in vitro.

**Conclusion:**

CYCS plays an oncogenic role in the pathophysiology of asthma, indicating that this gene may become a novel diagnostic biomarker and promising target of asthma treatment.

## 1. Introduction

Asthma (also known as bronchial asthma) is a long-term inflammatory condition of the lungs. With the rising incidence and mortality, asthma grows into a global health problem [1]. According to modern medicine, allergies, airway inflammation, airway hyperresponsiveness, airway remodeling [2], neuromodulation processes, and psychosocial variables are thought to be related to the pathophysiology of asthma [3, 4]. From the aspect of Chinese medicine, the pathophysiology of asthma is caused by “wind,” that is, phlegm blocking the lungs and phlegm stasis producing asthma, thus leading to inner disharmony. Increased airway reactivity associated with the above theory including numerous inflammatory cells, structural cells, and others can be fatal for asthma patients [5, 6]. The signs and symptoms of asthma contain shortness of breath, cough, chest tightness, and wheezing, which can be used to facilitate its diagnosis [7]. Currently, there is still a pressing need to uncover novel therapeutic targets for asthma patients.

The integration of bioinformatics and microarray technology has shown significant promise in evaluating the molecular and genetic pathways of malignant tumors, increasing carcinogenesis, development, and metastasis studies in recent decades [8]. Weighted gene coexpression network analysis (WGCNA) is a comprehensive and systematic biological technique for building network analysis to investigate gene-trait relationships. This mathematical concept was initially proposed in 2005 and the implemented as the “WGCNA package” in the R environment in 2008 [9]. WGCNA has been widely employed in recent years in a variety of domains, including the discovery of putative biomarkers from uveal melanoma [10], breast cancer [11], and adrenocortical carcinoma [12]. Researchers can apply WGCNA to investigate underlying relations between closely linked genes and find novel diagnostic or therapeutic targets in disease-associated gene clusters. So far, WGCNA has been seldom connected to the study of bronchial asthma.

As a result, this research tries to explore new therapeutic targets of asthma through WGCNA analysis, which will offer a fresh perspective on bronchial asthma research. First, we plan to identify differentially expressed genes (DEGs) from the GSE64913 dataset and then performed WGCNA. After targeting the key module, we will analyze its genes by protein-protein interaction (PPI) network, expression validation, and receiver operating characteristic (ROC) analysis to find the key gene related to asthma. These findings may help shed new light on asthma treatment.

## 2. Materials and Method

### 2.1. Asthma-Related Database Acquisition and Identification of DEGs

The asthma-related dataset GSE64913 was found and downloaded by National Center for Biotechnology Information (NCBI, https://www.ncbi.nlm.nih.gov/). The dataset included 28 asthma and 42 healthy samples. After that, the upregulated and downregulated DEGs in the samples were screened by the “limma” package of the R software, and *P* < 0.01, fold change (FC) > 1 (upregulation) or <1 (down-regulation) were set as the screening criteria, and the correlation heat map was drawn by the “pheatmap” package.

### 2.2. Enrichment Analysis on DEGs

After screening DEGs from the GSE64913 dataset, to explore the enrichment functions of these DEGs, we uploaded the sequence information of DEGs to the DAVID database, respectively. Then, Gene Ontology (GO) term and Kyoto Encyclopedia Gene Genome (KEGG) pathway enrichment analyses were applied on DEGs in this database, and the enrichment results with *P* < 0.05 were screened.

### 2.3. WGCNA Analysis

WGCNA has been widely applied to effectively investigate the relation between genome and clinical phenotype. This time, based on DEGs, we used WGCNA technology to construct a gene coexpression network. Specifically, a dendrogram of 70 samples in the GSE64913 dataset was constructed to determine the optimal soft threshold in the cowhite network. The genes in the samples were then grouped into different modules by cluster dendrogram. Finally, the correlation between different gene modules and samples was evaluated by the Pearson correlation coefficient.

### 2.4. Bioinformatics Analysis on the Genes in the Key Module

The Search Tool for the Retrieval of Interacting Genes (STRING) database (https://string-db.org/) and the Cytoscape tool were used to construct a PPI network of key module genes for analyzing the relationship between different genes. On this basis, the Cytohubba plug-in was applied to compute the degree value of each gene in the PPI network, and the top 10 were chosen to construct the PPI subnetwork and analyzed by KEGG enrichment analysis.

### 2.5. Expression Validation and ROC Prognostic Analysis of 10 Genes in Asthma

Next, we first analyzed the expressions of 10 genes in asthma and control groups. Then, ROC curve analysis was performed for 10 genes' prognostic value in asthma, with 1-specificity (true positive rate, TPR) as the *x*-axis and sensitivity (false positive rate, FPR) as the *y*-axis, and the corresponding area under curve (AUC) values and 95% confidence intervals (CI) of the genes were computed. When the AUC value was greater than 0.7, it indicated that the gene had a better predictive ability for the prognosis of asthma. Based on these data and previous research, CYCS was determined as the key gene for the next analysis.

### 2.6. Expression Analysis of CYCS in Human Tissues and Pan-Cancers

Genotype-Tissue Expression (GTEx) is one of the common public databases for performing bioinformatics analysis, which provides RNASeq data from tissues contributed by healthy people, often in conjunction with the The Cancer Gene Atlas (TCGA) database. Herein, the levels of the CYCS in normal tissues were observed based on GTEx and then the expressions of the hub gene in various tumor tissues in the TCGA database. After that, based on the GTEx and TCGA databases, the expressions of the CYCS in normal and cancer tissues were compared to judge the regulatory role of the hub gene on cancer development.

### 2.7. The Relation between CYCS and Immune Cells

TISIDB is a tumor immunity-related database that records 988 genes related to antitumor immunity. This time, we examined the correlation between 28 tumor-infiltrating lymphocytes (TILs) and hub gene in this database and drew the correlation heat map. Followed by, Spearman correlation analysis was applied to detect the correlation between hub gene and immunosuppressant, chemokine, and immune stimulants in the GSE64913 dataset. When *P* < 0.05, the obtained results were statistically significant.

### 2.8. Cell Culture

The human bronchial epithelial cell (16-HBE) was acquired from the Type Culture Collection, Chinese Academy of Sciences (Shanghai, China). The cells were grown in RPMI-1640 medium with 10% heat-inactivated fetal bovine serum (Hyclone), 100 mg/ml streptomycin, and 100 U/ml penicillin at 37°C with 5% CO_2_ in a humidified environment.

### 2.9. Cell Transfection

Two siRNAs against CYCS (si-CYCS #1, si- CYCS #2) and si-NC were synthesized from GenePharma (Shanghai, China). The CYCS mimics (over-CYCS #1, over-CYCS #2) and negative control mimic (over-NC) were designed by Ribobio (Guangzhou, China). As instructed, the abovementioned molecular synthesis was transfected into 16-HBE by Lipofectamine 2000 (Life Technologies).

### 2.10. qRT-PCR

TRIzol reagent (Invitrogen) was adopted to extract RNA from cell lines. The SuperScript RT kit (Invitrogen) was used to reverse transcribe 2 *μ*g of RNA for each sample. qRT-PCR was conducted by SYBR Premix Ex TaqTM (Takara, Japan). The relative expression level of target genes was computed by the 2^-*ΔΔ*Ct^ method.

### 2.11. Cell Counting Kit-8 (CCK-8) Assay

Cell proliferation was determined by CCK-8 assay kit (Beyotime, Shanghai, China). 16-HBE cells (5000 cells/well) were seeded in 96-well plates for 0, 24, 48, 72, or 96 hours after transfection. After that, each well was filled with 10 *μ*l of CCK-8 solution for 3 hours. A microplate reader (Bio-Tek, Winooski, VT) was used to measure absorbance at a wavelength of 450 nm.

## 3. Results

### 3.1. Identification and Analysis of DEGs Related to Asthma

We analyzed 70 samples from the GSE64913 dataset, and all genes associated with asthma progression were sequenced. Under the constraints of FC value and *P* value, 711 upregulated and 684 downregulated DEGs were screened (Figure 1(a)). Next, we performed GO term and KEGG pathway enrichment analysis for two kinds of DEGs, respectively. In GO terms, the upregulated DEGs were enriched in purine-containing compound salvage, skin development, positive regulation of mitochondrion organization (biological process, BP), mitochondrial membrane, organelle inner membrane, cornified envelope, mitochondrial inner membrane (cell components, CC), cadherin binding, intramolecular transferase activity, and phosphotransferases (molecular function, MF) (Figure 1(b)). In KEGG, we got 30 pathways enriched by upregulated DEGs, such as apoptosis, Parkinson's disease, diabetic cardiomyopathy, colorectal cancer, estrogen signaling pathway, and p53 signaling pathway (Figure 1(c)). Similarly, according to Figure 1(d), it could be seen that the downregulated DEGs were related to the cellular response to interferon-gamma, regulation of RNA splicing in BP, MHC protein complex, MHC class II protein complex and others in CC, and MHC class II protein complex binding in MF. In addition, the enrichment results of KEGG showed the enrichment pathways of downregulated DEGs included antigen processing and presentation, influenza A, and other pathways (Figure 1(e)).

### 3.2. Identification of the Brown Module in WGCNA

Expression data of 1395 DEGs were extracted from GSE64913 and used to perform WGCNA (Figure 2(a)). By setting the soft threshold power to 20 (unscaled *R* = 0.85, Figure 2(b)), we obtained seven modules (Figures 2(c) and 2(d)) and constructed the corresponding cluster dendrogram and eigengene adjacency heat map. Among them, there are nonaggregated genes in the gray module, which are not analyzed. From the heat map of module-trait correlations, we found the brown module had the highest correlation value with a Pearson correlation coefficient of 0.598, *P* = 4.7*e* − 08, so we identified the brown module as the key module (Figure 2(e)).

### 3.3. PPI Network and KEGG Enrichment Pathway Analysis on the Genes in the Brown Module

We considered the brown module to be the key module related to asthma and then analyzed it in detail. The key module contained 78 genes, and the interactions of genes were shown in the PPI network in Figure 3(a). Then, according to the Cytohubba algorithm, the degrees of the genes in the PPI network were sorted (Figure 3(b)), and the genes with the top 10 degree values were selected to construct a subnetwork. As shown in Figure 3(c), the top 10 genes were CD44, CYCS, DDIT3, SFN, PMAIP1, LDHA, FKBP5, ANXA8, ATF4, and S100A2. To explore the potential biological functions of the top10 genes, KEGG analysis was performed, and the enrichment pathways were shown in Figure 3(d), mainly p53 signaling pathway, apoptosis, lipid and atherosclerosis, Parkinson disease, and other pathways.

### 3.4. Expression Validation and Prognostic Value Analysis on the above 10 Genes

In the expression analysis of 10 genes in the asthma and control groups, it was found that the 10 genes were generally low-expressed in the control group and highly expressed in the asthma group (Figure 3(e)). Hence, we inferred these 10 genes played an oncogenic role in the progression of asthma. In the subsequent ROC curve analysis results, according to the AUC value, we found that ATF4 (AUC = 0.869) had the strongest prognostic ability in asthma patients, followed by FKBP5 (AUC = 0.838), CD44 (AUC = 0.787), SFN (AUC = 0.766), S100A2 (AUC = 0.748), and CYCS (AUC = 0.714). The AUC values of the left 4 genes were all less than 0.7, indicating a low accuracy in predicting the prognosis of asthma patients (Figure 3(f)). Combined with the previous research, CYCS was chosen as the key gene for the next study.

### 3.5. Expression and Immunoassay of CYCS in Human Tissues and Pan-Cancer

By using GTEx database, we found that the atrial appendage, left ventricle, cell-EBV-transformed lymphocytes, and muscle-skeletal tissues all had greater levels of CYCS gene expression (Figure 4(a)). Next, we also examined the expression of CYCS in various tumor tissues in the TCGA database (Figure 4(b)). Furthermore, combined with the TCGA and GTEx databases, we found that that the expression of CYCS was generally higher in tumor tissues (Figure 4(c)). In the immune analysis of CYCS, we examined the association between this gene and 28 TILs through the TISIDB database and found that the association between CYCS and TILs varied in different cancer types (Figure 4(d)). Spearman's analysis showed that CTCS was inversely correlated with IDO1 and TGFBR1 in immunosuppressants (Figure 4(e)). Among chemokines, CYCS was positively correlated with CCL18 and CCL23 and negatively correlated with CXCL1, CXCL2, CXCL3, and CXCL8 (Figure 4(f)). Among immune stimulants, CYCS was positively associated with HHLA2, while negatively with IL6 and MICB (Figure 4(g)).

### 3.6. The Effects of CYCS Knockdown and Overexpression on the Proliferation of 16-HBE Cells

CYCS was knocked down in human bronchial epithelial cell 16-HBE by transfection with si-CYCS #1 and si-CYCS #2. Knockdown efficiency was confirmed using qRT-PCR, and si-CYCS #2 had a better knockdown effect (Figure 5(a)). Next, we examined the effect of CYCS knockdown on cell proliferation in 16-HBE cells. As shown in Figure 5(b), si-CYCS #2 significantly promoted the cell proliferation. Besides, CYCS was then overexpressed in 16-HBE cells by transfection of over-CYCS #1 and over-CYCS #2, and over-CYCS #1 had better overexpression efficiency, confirmed by qRT-PCR (Figure 5(c)). As shown in Figure 5(d), over-CYCS #1 significantly inhibited the proliferation of cells.

### 3.7. The Cytokines Are Positively Regulated by CYCS

Next, we transfected si-CYCS #1, si-CYCS #2, over-CYCS #1, and over-CYCS #2 into 16-HBE cells to observe the relation between CYCS and chemokines (CCL-17), inflammatory cytokines (IL-5, IL-8, and COX-2) in human bronchial epithelial cell lines [13]. We found that the levels of cytokines were concomitantly decreased in 16-HBE cells with si-CYCS (Figures 5(e)–5(h)). Moreover, 16-HBE cells were then transfected with over-CYCS #1 and over-CYCS #2 to elevate CYCS expression. The expression levels of cytokines were subsequently increased in 16-HBE cells. In addition, cytokine expression was mostly elevated in the over-CYCS #2 group (Figures 5(i)–5(l)).

## 4. Discussion

As a complex disease, asthma has a confusing pathological mechanism. In recent years, people have carried out a series of explorations on the pathogenesis of asthma by using clinical phenotypes, combining corresponding molecular tools and targeting monoclonal antibodies. After research, some scholars believe that the most common cause of asthma exacerbation may be viral respiratory infections [14, 15], especially human rhinovirus. Presently, long-acting beta-agonists and targeted drug therapy are applied to prevent asthma progressions, such as anti-IgE and anti-IL-5. As asthma often presents with obvious heterogeneous symptoms, Walsh believes that IL-4, IL-5, and IL-13 have considerable potential in the treatment of asthma, and anti-IL-5 monoclonal antibody prevents disease exacerbation in asthmatic patients [16]. Francisco believes that aerobic exercise can improve nocturnal exacerbation of asthma symptoms, especially in children [17]. In addition, several studies have discussed biomarkers of asthma that can be obtained from a variety of biological sources, including exhaled air, serum, and urine [18, 19]. Herein, we aimed to screen a hub gene for asthma diagnosis and treatment from pertinent database by a series of bioinformatics analyses and functional experiments.

GO and KEGG enrichment analyses are frequently used in bioinformatics research, which allows for the extraction of valuable information, such as gene biological characteristics, gene regulation relationships, and gene function and meaning. In this asthma study, we identified 711 upregulated and 684 downregulated DEGs from the GSE64913 dataset, and they were mainly enriched in purine-containing compound salvage, skin development, gluconeogenesis, Parkinson disease, diabetic cardiomyopathy, colorectal cancer, influenza A, and others involved in the regulation of asthma pathogenesis. For example, some skin diseases are associated with some allergens like isocyanates that may also contribute to asthma [20]. Skin may also be an important site for asthma attacks, and the impaired skin barrier function may lead to the invasion of allergens, thereby triggering Th2-like sensitization and asthma attacks [21, 22]. Gluconeogenesis refers to the process of converting nonsugar compounds into glucose or glycogen, which helps maintain the body's balance [23]. FBP1 is one of the rate-limiting enzymes in gluconeogenesis. Hu et al. found that FBP1 could induce asthma cell apoptosis by inhibiting the NRF2 pathway [24]. Besides, several studies have shown that influenza A virus infection in asthmatics can cause serious complications, such as plastic bronchitis [25]. These results demonstrate that these DEGs meet the condition for the asthma analysis.

The purpose of WGCNA in bioinformatics analysis is to show the coexpression relationship between genes, which can improve the accuracy of analyzing the association between genes and diseases. Herein, we acquired the key module-brown module (78 genes) highly associated with asthma based on the WGCNA algorithm. Then, according to the STRING database and Cytoscape software, a PPI network of key modules was constructed. According to the value of the degree in the network, 10 key genes related to asthma were chosen for the key gene identification, namely, CD44, CYCS, DDIT3, SFN, PMAIP1, LDHA, FKBP5, ANXA8, ATF4, and S100A2. Next, we performed KEGG enrichment analysis on these 10 genes and obtained 10 significantly correlated pathways, namely, p53 signaling pathway, nonalcoholic fatty liver disease, apoptosis, lipid and atherosclerosis, Parkinson disease, prion disease, amyotrophic lateral sclerosis, Alzheimer disease, colorectal cancer, and glucagon signaling pathway. Among them, the p53 signaling pathway is involved in tumor progression, such as gastric cancer [26], breast cancer [27], and pancreatic cancer [28]. Nonalcoholic fatty liver disease is associated with insulin resistance and genetic susceptibility and can cause hyperlipidemia, liver fibrosis, and liver cirrhosis and atherosclerosis [29]. Some studies have found that abnormal expression of CD44 is associated with liver disease progression in patients with nonalcoholic fatty liver disease [30]. So far, the association between the above KEGG pathways in asthma has not been discovered.

Afterward, we examined the expressions of 10 key genes in asthma and control samples and found that 10 genes were generally highly expressed in asthma samples, indicating that these genes had a promoting effect on the pathogenesis of asthma. The results of subsequent ROC analysis also showed that ATF4, FKBP5, CD44, SFN, S100A2, and CYCS had a higher prognostic predictive ability. In previous studies, the first five genes have been reported to be related to asthma development. Guo et al. confirmed that PERK-ATF4-CHOP signaling was linked to asthmatic airway inflammation [31]. Alsaffar et al. analyzed the association between FKBP5 gene polymorphisms and asthma patients by sequencing and found that the FKBP5 variant could predict asthma susceptibility [32]. CD44 is a receptor for hyaluronic acid [33], which can interact with ligands, such as osteopontin, collagen, and matrix metalloproteinases. In addition, CD44 is one of the eosinophil surface proteins, and its activation state has been confirmed to be associated with the onset of asthma [34]. Moreover, Hachim et al. found that the SFN gene was associated with cell cycle and proliferation in asthma cell experiments, and the gene was upregulated in asthmatic bronchial epithelial cells [35]. S100A2, a member of the S100 protein family, is involved in the regulation of many cellular processes and can play a role in many physiological processes. For instance, Poachanukoon et al. discovered the S100A2 gene in samples from asthma patients [36]. The relation between CYCS and asthma mechanism has not been explored. Thus, CYCS gene was selected as the research target.

As a central component of the electron transport chain in mitochondria, CYCS has been reported to be involved in the initiation of cell apoptosis [37]. The binding of CYCS to Apaf-1 triggers the activation of caspase-9, which accelerates cell apoptosis by activating other caspases. Other studies also suggest that mutations in CYCS are associated with autosomal dominant nonsyndromic thrombocytopenia [38]. To investigate the biological properties of CYCS in the pathogenesis of asthma, we examined the expressions of this gene in pan-cancers using the TCGA and GTEx databases. The obtained results showed that this gene was generally highly expressed in tumor tissues, and it was inferred that this gene could act as a tumor-promoting factor in cancer, which was testified by the following functional experiments. The knockdown of CYCS expression in the human bronchial epithelial cell line 16-HBE promoted cell proliferation. Conversely, cell proliferation is inhibited by its overexpression.

Afterward, we also validated the relationship between CYCS and immunosuppressants, chemokine, and immunostimulants in the dataset GSE64913 [39]. It was found that CYCS was negatively correlated with IDO1, TGFBR1, CXCL1, CXCL2, CXCL, CXCL8, IL6, and MICB immune factors, while positively correlated with CCL18, CCL23, and HHLA2 immune factors. These results indicate CYCS might have a functional role in immune cells. Tumor microenvironment (TME) is a complex and comprehensive system, including tumor cells, surrounding immune and inflammatory cells, and various cytokines and chemokines [40]. Recently, researchers try to find new therapies for cancers, that is called immunotherapy. In our experimental results, qPCR experiments showed that the levels of cytokines in 16-HBE cells decreased with the up- and downregulated changes of CYCS, indicating that cytokines (CCL-17, IL-5, IL-8, and COX-2) are positively regulated by CYCS. In recent studies on asthma, anti-IL-5 therapy has been shown to slow the exacerbation of eosinophilic severe asthma, IL-8 antagonism can be used in the treatment of asthma, and COX-2 is also associated with allergic asthma [41–43]. This findings might offer new directions for the development of asthma immunotherapy.

In conclusion, our study confirms the promoting role of CYCS in asthma samples and its positive relation with cytokines. These findings indicate that CYCS might be a new diagnostic indicator and promising target for asthma immunotherapy. However, the direct link between miRNA and mRNA will be performed on the same patients' samples in the future study. The exact mechanism of CYCS still needs investigating, which will be conducted in our further study.

## Figures and Tables

**Figure 1:** Identification and functional enrichment analysis of DEGs in the GSE64913 dataset. (a) 1395° cluster heat map, blue represents the asthma group, and orange represents the control group. Red refers to upregulation, and blue refers to downregulation. (b, c) GO (including BP, CC, and MF) and KEGG enrichment analysis of upregulated DEGs. (d, e) GO and KEGG enrichment analysis of downregulated DEGs.

**Figure 2:** WGCNA analysis of DEGs in the GSE64913 dataset. (a) Sample clustering to detect outliers. (b) Scale-free topology model (top) and average connectivity (bottom) for finding the soft-threshold capability. Power is 20. (c) Hierarchical dendrogram showing coexpression modules recognized by WGCNA. Each leaf on the tree represents a gene. The main tree is divided into 7 modules according to the eigengene calculations, and each module is highlighted with a different color. (d) Clustering of all modules. (e) Heat map showing the relationship between different modules and clinical features.

**Figure 3:** Screening of candidate key genes, expression level analysis, and ROC diagnostic value analysis. (a) PPI network graph of genes in brown modules, including 40 nodes and 45 edges. (b) Degree ranking of genes by Cytohubba software. (c) PPI network of the 10 genes with the highest height values. (d) KEGG enrichment analysis of the top 10 genes. (e) Expression levels of 10 genes, listed by ANXA8, ATF4, CD44, CYCS, DDIT3, FKBP5, LDHA, PMAIP1, S100A2, and SFN. (f) ROC analysis on the top 10 genes. The abscissa is 1-specificity (FPR), and the ordinate is sensitivity (TPR). The closer the curve is to the upper left corner, the higher the prediction accuracy. ^∗^*P* < 0.05, ^∗∗^*P* < 0.01, and ^∗∗∗^*P* < 0.001.

**Figure 4:** Validation of CYCS expression in tumors and analysis of immune levels. (a) Expression of CYCS in human tissues. (b) CYCS expression in TCGA tumors. (c) Comparative analysis of CYCS expression levels in normal and tumor tissues. (d) Heat map of the correlation analysis between CYCS and immune infiltration levels in pan-cancer. (e) Correlation analysis between CYCS and immunosuppressants. (f) Correlation analysis between CYCS and chemokines. (g) Correlation analysis between CYCS and immunostimulants. ^∗^*P* < 0.05, ^∗∗^*P* < 0.01, and ^∗∗∗^*P* < 0.001.

**Figure 5:** The differential expression of CYCS regulates the proliferation and cytokine expression levels of 16-HBE cells. (a) Confirmation of knockdown transfection efficiency of si-CYCS #1 and si-CYCS #2 using qRT-PCR. (b) Si-CYCS #2 promotes cell proliferation in 16-HBE cells. (c) The transfection efficiency of CYCS #1 and CYCS #2 overexpression was confirmed using qRT-PCR. (d) Over-CYCS #1 inhibits cell proliferation of 16-HBE cells. (e–h) Expression of CCL-17, IL-5, IL-8, and COX-2 expressions in cells with si-CYCS. (i–l) CCL-17, IL-5, IL-8, and COX-2 expressions in over-CYCS cells. ^∗^*P* < 0.05, and ^∗∗^*P* < 0.01.

## Data Availability

The datasets used and/or analyzed during the current study are available from the corresponding author on reasonable request.
